# Epidemiological Investigation and Risk Factor Analysis of Acute Hemorrhagic Conjunctivitis in Huangshi Port District, Huangshi City

**DOI:** 10.1155/2022/3009589

**Published:** 2022-05-02

**Authors:** Juan Liu, Hui Zhang

**Affiliations:** ^1^Department of Science and Education, Huangshi Central Hospital, Affiliated Hospital of Hubei Polytechnic, Edong Healthcare Group, Hubei Key Laboratory of Kidney Disease Pathogenesis and Intervention, No. 141 Tianjin Road, Huangshi, Hubei 435000, China; ^2^Technical Service Center, Kunming Center for Disease Control and Prevention, Kunming, Yunnan 650034, China

## Abstract

**Objective:**

This study is aimed at investigating the epidemiology and risk factors of acute hemorrhagic conjunctivitis (pinkeye) in Huangshi Port District of Huangshi City.

**Methods:**

A total of 593 cases of acute hemorrhagic conjunctivitis from January 2019 to December 2021 were selected as the observation group. The epidemiological characteristics (age of onset, season, occupation, clinical manifestations, and etiological characteristics) were analyzed. A total of 425 healthy subjects (nonacute hemorrhagic conjunctivitis) were selected as the control group. The general data of the two groups were compared, and the risk factors affecting the occurrence of acute hemorrhagic conjunctivitis were analyzed by logistic regression.

**Results:**

The onset age of acute hemorrhagic conjunctivitis was mainly concentrated in 0-20-year-old and 60-year-old age groups, and the onset season was mainly concentrated in April to August, with the highest incidence in May. The proportions of middle school students and workers in patients with acute hemorrhagic conjunctivitis were higher than those of other occupations (both *P* < 0.05). Ocular conjunctival congestion, tingling, and foreign body sensation were the main clinical manifestations of patients with acute hemorrhagic conjunctivitis. Among the 593 conjunctival swab samples collected in this study, the positive rates of HEV70 and CVA24v were higher than those of adenovirus nucleic acid (both *P* < 0.05). The proportion of people aged ≤40 years old, male, working outdoors, using potable water equipment, contact history of patients with acute conjunctivitis, history of chemical substances entering eyes, combined with immune system diseases, and public toilet utilization rate ≥ 1 times/d in the observation group was higher than that in the control group (all *P* < 0.05), and the proportion of people washing hands before eating and after toilet was lower than that in the control group (*P* < 0.05). Multiple logistic regression analysis showed that working place outdoors, use of potable water equipment, contact history of patients with acute conjunctivitis (all *P* < 0.05), and use of public toilets ≥ once a day were risk factors for the occurrence of acute hemorrhagic conjunctivitis, and washing hands before eating and after toilet was a protective factor (*P* < 0.05).

**Conclusion:**

The onset age of acute hemorrhagic conjunctivitis was mainly concentrated in 0-20-year-old and 60-year-old age; the onset season was mainly concentrated in summer and autumn; adenovirus is the main pathogenic bacteria; ocular conjunctivitis congestion, tingling, and foreign body sensation were the main clinical manifestations; working place outdoors, use of potable water equipment, contact history of patients with acute conjunctivitis (all *P* < 0.05), and use of public toilets ≥ once a day were risk factors for the occurrence of acute hemorrhagic conjunctivitis, while washing hands before eating and after toilet was a protective factor.

## 1. Introduction

Eyeball is an important organ of the human body. Once eyeball infection occurs, it will damage the vision of patients. Acute hemorrhagic conjunctivitis is a self-limited eye infectious disease caused by enterovirus 70 (EV70), coxsackievirus A24 variant (CVA24v), and adenovirus (Adv) in microribonucleic acid virus, commonly known as “pinkeye.” The patient is mainly manifesting symptoms such as eye pain, redness, and increased eye secretion and conjunctival congestion [1, 2]. Acute hemorrhagic conjunctivitis is characterized by rapid onset and strong infectivity, and there have been global pandemics and many local outbreaks of this disease. At present, due to effective prevention and control, no serious clusters of cases of this disease have been reported in China, and the incidence is decreasing year by year. Nevertheless, sporadic epidemics still occur in some areas of China, so the analysis of local epidemiology plays an important role in the later prevention [3, 4]. Relevant reports pointed out that conjunctivitis can spread to the cornea and cause some degree of visual impairment. Targeted intervention for various high-risk groups can reduce the incidence of acute hemorrhagic conjunctivitis. Therefore, it is very important to analyze the risk factors affecting the occurrence of this disease [5]. Clinical data show that poor sanitation is the main cause of the occurrence of acute hemorrhagic conjunctivitis, and the patient's immune function is also closely related to the occurrence of the disease, but there is no conclusion on the risk factors affecting the occurrence of the disease [6]. Therefore, the purpose of this study is to analyze the epidemiology of acute hemorrhagic conjunctivitis in this region and the risk factors affecting its occurrence, so as to provide reference for the clinical prevention and treatment of the disease.

## 2. Materials and Methods

### 2.1. Clinical Data

Our data came from the National Disease Control and Prevention Information System, in which the infectious disease report card made statistics of clinical diagnosis and laboratory diagnosis by current address and onset date. Population data came from the National Basic Information System. A total of 593 cases of acute hemorrhagic conjunctivitis in Huangshi Port District, Huangshi City, from January 2019 to December 2021 were selected as the observation group, and 425 healthy subjects (nonacute hemorrhagic conjunctivitis) were selected as the control group. Inclusion criteria were as follows [7]: (1) the observation group met the diagnostic criteria; according to the standard of Chinese health industry-acute hemorrhagic conjunctivitis, the clinical cases met the following conditions: (1) had an epidemiological history; (2) typical clinical symptoms and obvious signs; and (3) conjunctival cytological examination showed that the nucleus reaction of the diaphragma sella was dominant. (2) Complete clinical data. Exclusion criteria are as follows: (1) patients with nosocomial infection; (2) pregnant or lactating women; and (3) patients with other types of conjunctivitis.

### 2.2. Methods

#### 2.2.1. Clinical Data Collection

General information questionnaire was used to collect the general information of the subjects, including residence, season of onset, occupation, clinical manifestations, gender (male vs. female), age (≤40 vs. >40), workplace (outdoor vs. indoor), education level (junior high school and below vs. senior high school and above), use of potable water equipment, smoking, and drinking. Smoking meant averaged 1 cigarette per day and lasting for more than 6 months. Drinking was defined as alcohol intake ≥ 40 g/d for men and ≥20 g/d for women and duration ≥ 6 months.

#### 2.2.2. Etiological Analysis

The conjunctiva of the patient was wiped with a sterile cotton swab, and the specimen was stored in 2 ml virus specimen transport solution. Viral RNA and DNA were extracted using Qiagen's QIAamp MinElute Virus Spin Kit. The primers were synthesized by Shanghai Sangon (China): (1) HEV70: upstream primer: 5′-AGGGATTCACCAGACATTGG-3′ and downstream primer: 5′-ATTTTCCACCAGGCACTCTG-3′, product size: 242 bp; (2) CVA24v: upstream primer: 5′-GTGAGTGCTTGCCCAGATTT-3′ and downstream primer: 5′-CTCCACTAGAGCGGTGTG-3′, product size: 184 bp; and (3) adenovirus: upstream primer: 5′-GCCSCARTGGKCWTACATGCACATC-3′A and downstream primer: 5′-CAGCACSCCICGRATGTCAAA-3′, product size: 301 bp. HEV70 and CVA24v were amplified using the One-Step RNA PCR Kit of the Qiagen company, and adenovirus nucleic acid was amplified using the GoTaq Green Master Kit of the Promega company. The amplified products were electrophoresed on 2% agarose containing ethidium bromide and observed under the automatic gel imaging system.

### 2.3. Observational Indices

(1) The epidemiological characteristics of acute hemorrhagic conjunctivitis, including onset age, season, occupation, and clinical manifestations, were analyzed. (2) The general data of the observation group and the control group were compared to analyze the risk factors affecting the occurrence of acute hemorrhagic conjunctivitis.

### 2.4. Statistics Process

SPSS22.0 software was used for data processing. The counting data were expressed with percent, and the *χ*^2^ test was used for intergroup comparison. The measurement data were expressed by $\bar{x}\pm s$ after normal test, and *t*-test was used for intergroup comparison. All our data were verified before *t*-test, and statistical analysis was conducted only after they met the conditions. Multivariate logistic regression was used to analyze the risk factors of acute hemorrhagic conjunctivitis. GraphPad Prism 5 was used for graphing. *P* < 0.05 indicated that the difference was statistically significant.

## 3. Results

### 3.1. Epidemiological Characteristics

A total of 593 cases of AHC were reported from 2019 to 2021.The reported incidence was 7.45 per 10 000 cases in 2019, 8.67 per 10 000 cases in 2020, and 8.44 per 10 000 cases in 2021. No deaths were reported.

### 3.2. Seasonal Distribution of Acute Hemorrhagic Conjunctivitis

The onset season of acute hemorrhagic conjunctivitis was mainly concentrated from April to August, with the highest incidence in May (Figure 1).

### 3.3. Incidence Maps

The number of reported cases in different administrative areas of Yellowstone Port District from 2019 to 2021 is as follows: Shenjiying Street: 99, 16.69%; Huangshi Port Street: 102, 17.20%; Hongqiqiao Street: 115, 19.39%; Shengyang Port Street: 129, 21.75%; and Jiangbei Management District: 148, 24.96%.

### 3.4. Age Distribution of Acute Hemorrhagic Conjunctivitis

The age of onset of acute hemorrhagic conjunctivitis was mainly 0-20 years old and 60 years old (Figure 2).

### 3.5. Gender Distribution

A total of 351 male cases and 242 female cases were reported in Huangshi Port District from 2019 to 2021. The male to female ratio was 1.45 : 1. Male cases were more than female cases, and the difference was statistically significant (*X*^2^ = 50.223, *P* < 0.001).

### 3.6. Occupational Distribution of Acute Hemorrhagic Conjunctivitis

The proportion of middle school students and workers in patients with acute hemorrhagic conjunctivitis was higher than that of other occupations (*P* < 0.05, Figure 3).

### 3.7. Analysis of Clinical Manifestations of Acute Hemorrhagic Conjunctivitis

Ocular conjunctival congestion, tingling, and foreign body sensation were the main clinical manifestations of patients with acute hemorrhagic conjunctivitis (Figure 4).

### 3.8. Analysis of Etiological Characteristics of Acute Hemorrhagic Conjunctivitis

Among the 593 conjunctival swab samples collected in this study, the detection rate of HEV70 and CVA24v was higher than the positive rate of adenovirus nucleic acid (both *P* < 0.05, Table 1).

### 3.9. Univariate Analysis of Factors Affecting the Occurrence of Acute Hemorrhagic Conjunctivitis

The proportion of people aged ≤40 years old, male, working outdoors, using potable water equipment, contact history of patients with acute conjunctivitis, history of chemical substances entering eyes, combined with immune system diseases, and public toilet utilization rate ≥ 1 times/d in the observation group was higher than that in the control group (all *P* < 0.05), and the proportion of people washing hands before eating and after toilet was lower than that in the control group (*P* < 0.05, Table 2).

### 3.10. Multivariate Analysis of Factors Affecting the Occurrence of Acute Hemorrhagic Conjunctivitis

Outdoor working place, use of potable water equipment, contact history of patients with acute conjunctivitis, and public toilet utilization rate ≥ 1 times/d were the risk factors for the occurrence of acute hemorrhagic conjunctivitis (all *P* < 0.05), and hand washing before eating and after toileting was a protective factor (*P* < 0.05,Table 3).

## 4. Discussion

Acute hemorrhagic conjunctivitis, commonly known as pinkeye, is an acute viral eye disease that has been prevalent in the world in the past 40 years. The disease has a short incubation period. Simultaneous or sequential onset of both eyes can occur within a short time after contact with the source of infection, and patients are often accompanied by foreign body sensation, photophobia, and other eye irritation symptoms. In this study, the clinical symptoms of the included patients were statistically analyzed, and it was found that ocular conjunctival congestion, tingling, and foreign body sensation were the main clinical manifestations of patients with acute hemorrhagic conjunctivitis, which was consistent with relevant reports [8]. This basically is because that obstruction of blood circulation to the conjunctiva after infection with pathogenic bacteria leads to symptoms such as conjunctival congestion and tingling. Due to the strong infectivity of the disease, the population is generally susceptible to it. If there is a large-scale epidemic, it may cause a large medical burden and social and economic losses, and in serious cases, it may lead to the spread of acute hemorrhagic conjunctivitis among countries [9]. Relevant studies indicate that the impact of acute hemorrhagic conjunctivitis on social and medical care can be alleviated by analyzing the epidemiological characteristics of the disease and providing targeted intervention to the relevant high-risk groups [10, 11]. In recent years, there have been many reports on the prevalence of acute hemorrhagic conjunctivitis. However, due to the differences in demographic characteristics in different regions, this study was conducted to investigate the epidemiological and etiological characteristics of acute hemorrhagic conjunctivitis in local region.

Relevant reports point out that acute conjunctivitis is a seasonal infectious disease which occurs mostly in summer [12]. Our study also found that the onset season of acute hemorrhagic conjunctivitis was mainly concentrated in April to August, with the highest incidence in May. This result was not significantly different from the above results, indicating that the onset season of the disease in this region was consistent with other regions. This may also be related to the fact that HEV70 and CVA24v are suitable for survival and transmission in warm and humid environment [13]. Acute hemorrhagic conjunctivitis is mainly caused by HEV70 and CVA24v infection. Studies in China have found that HEV70 and CVA24v are the main pathogenic bacteria of acute hemorrhagic conjunctivitis [14, 15]. Some serotypes of adenovirus have also been reported to cause the disease [16, 17]. In conjunctival swab samples collected in the present study, the detection rate of HEV70 and CVA24v was higher than the positive rate of adenovirus nucleic acid, indicating that HEV70 and CVA24v were still the main pathogenic bacteria of this disease, which is consistent with the above research results. Our study found that the onset age of acute hemorrhagic conjunctivitis was mainly concentrated in 0-20-year-old and 60-year-old age group, indicating that younger or older patients have a higher risk of acute hemorrhagic conjunctivitis. This is mainly related to the decreased body resistance of patients. Poor hygiene or lifestyle in younger or older patients may also influence the occurrence of acute hemorrhagic conjunctivitis. Relevant reports pointed out that the probability of acute hemorrhagic conjunctivitis is not the same in different occupations [18]. The results of our study showed that the proportion of middle school students and workers in patients with acute hemorrhagic conjunctivitis was higher than that of other occupations, indicating that the probability of students suffering from acute hemorrhagic conjunctivitis was higher, which was related to the high aggregation rate of school population.

The transmission route of acute hemorrhagic conjunctivitis is also a research hotspot. Clinical data show that the main transmission routes of the disease are the hands, towel, and handkerchief with eye secretion. Research points out that at present, acute hemorrhagic conjunctivitis is easy to be popular in the area with dense population and poor sanitary conditions [19, 20]. The present study found that the proportion of patients who were aged ≤40 years old, male, working outdoors, using portable water equipment, having contact history with patients with acute conjunctivitis, having history of chemical substances entering eyes, complicated with immune system diseases, and using public toilets ≥ 1 time/d in the observation group was higher than that in the control group, and the proportion of people who washed their hands after using the toilet and before eating was lower than that in the control group. It indicated that the occurrence of acute hemorrhagic conjunctivitis may be related to the use of portable water equipment. Further analysis of this study found that outdoor working place, use of portable water equipment, contact history of patients with acute conjunctivitis, and use of public toilets ≥ 1 time/d were risk factors for the occurrence of acute hemorrhagic conjunctivitis, while washing hands after using the toilet and before eating was a protective factor. It is suggested that the incidence of acute hemorrhagic conjunctivitis may be reduced by reducing the rate of using portable water equipment, isolating patients, strictly disinfecting public areas such as public toilets, and promoting the necessity of hand washing after toileting and before eating. The reason is that acute hemorrhagic conjunctivitis can be induced by contacting the secretion of diseased eyes by shaking hands and then rubbing their eyes with their contacted hands. In conclusion, working place outdoors, using portable water equipment, contact history of patients with acute conjunctivitis, and the rate of public toilet use ≥ 1 times/d were risk factors, while washing hands after toileting and before eating was a protective factor.

Schools are places with high incidence of infectious diseases, and clinical data show that nearly 70% of public health emergencies in China occur in schools, and the transmission rate of various infectious diseases in schools is quite high. Some scholars pointed out that the probability of suffering from acute hemorrhagic conjunctivitis in junior students is much higher than that in senior patients [21]. Our study found that the disease detection rate of 0-10-year-old patients ranked the second in the whole age group, which may be related to the poor personal hygiene awareness of students. They had low awareness of red eye disease and would not pay attention to their own disinfection and cleaning after contacting patients with red eye disease, so the occurrence of the disease was related to age. Further analysis in this study found that the age of patients was not a risk factor for the occurrence of the disease, which may be related to the excessively high age demarcation line in this study. Therefore, this study is expected to further analyze the correlation between age and the occurrence of this disease. The incidence of acute hemorrhagic conjunctivitis was higher in patients with contact ophthalmic examination [22]. When patients perform contact ophthalmic examination, the integrity of the eye mucosa was destroyed, which provided a favorable path for pathogenic microorganisms and increased the contact time between the eyeball and the external environment and external viruses, thus increasing the chance of infection. However, the results of this study showed that contact ophthalmic examination was not a risk factor for the occurrence of acute hemorrhagic conjunctivitis, which was inconsistent with the results of the above study. This may be related to the small number of patients with neutral contact ophthalmic examination in this study, so further analysis should be conducted later.

In conclusion, the onset age of acute hemorrhagic conjunctivitis was mainly concentrated in 0-20-year-old and 60-year-old age groups, and the onset season was mainly concentrated in summer and autumn. HEV70 and CVA24v were the main pathogenic bacteria, and the main clinical manifestations were ocular conjunctivitis congestion, pain, and foreign body sensation. The risk factors for the occurrence of acute hemorrhagic conjunctivitis were working place outdoors, using portable water equipment, contact history of patients with acute conjunctivitis, and the rate of public toilet use ≥ 1 times/d, while washing hands after toileting and before eating was a protective factor.

## Figures and Tables

**Figure 1:** Seasonal distribution of acute hemorrhagic conjunctivitis.

**Figure 2:** Age distribution of acute hemorrhagic conjunctivitis.

**Figure 3:** Occupational distribution of acute hemorrhagic conjunctivitis.

**Figure 4:** Analysis of clinical manifestations of acute hemorrhagic conjunctivitis.

**Table 1:** Analysis of etiological characteristics of acute hemorrhagic conjunctivitis (case, %).

Pathogenic bacteria	Number of cases	Constituent ratio
HEV70	217	36.59
CVA24v	142	23.95
Adenovirus	2^∗^^#^	0.34

Note: compared with HEV70, ^∗^*P* < 0.05; compared with CVA24v, ^#^*P* < 0.05.

**Table 2:** Univariate analysis of factors affecting the occurrence of acute hemorrhagic conjunctivitis (case, %).

Factor		Observation group (*n* = 593)	Control group (*n* = 425)	*χ* ^2^	*P*
Age	≤40 years old	308 (51.94)	173 (40.71)	12.534	<0.001
	>40 years old	285 (48.06)	252 (59.29)		
Gender	Male	351 (59.19)	229 (53.88)	50.223	<0.001
	Female	242 (40.81)	364 (85.65)		
Working place	Outdoor	319 (53.79)	254 (59.76)	14.266	<0.001
	Indoor	274 (46.21)	339 (79.76)		
Educational level	Junior high school or below	442 (74.54)	336 (79.06)	2.810	0.094
	Senior high school or above	151 (25.46)	89 (20.94)		
Use of potable water equipment		194 (32.72)	87 (20.47)	53.395	<0.001
Contact history of patients with acute conjunctivitis		531 (89.54)	147 (34.59)	336.140	<0.001
History of ocular trauma		93 (15.68)	85 (20.00)	0.423	0.515
History of eye surgery		32 (5.40)	19 (4.47)	3.463	0.063
History of chemical substances entering the eyes		44 (7.42)	15 (3.53)	15.000	<0.001
History of contact ophthalmic examination		52 (8.77)	49 (11.53)	0.097	0.755
Combined with other infectious diseases		31 (5.23)	19 (4.47)	3.007	0.083
Combined with immune system diseases		66 (11.13)	37 (8.71)	8.942	0.003
Washing hand before eating and after toileting		317 (53.46)	376 (88.47)	12.084	0.001
Smoking		125 (21.08)	99 (23.29)	3.721	0.054
Drinking		103 (17.37)	91 (21.41)	0.887	0.346
Public toilet utilization rate ≥ 1 times/d		239 (40.30)	117 (27.53)	59.742	<0.001

**Table 3:** Multivariate analysis of factors affecting the occurrence of acute hemorrhagic conjunctivitis (case, %).

Index	*β*	SE	Wald *χ*^2^	OR	95% CI	*P*
Age	0.538	0.321	2.809	1.713	0.913~3.213	0.094
Gender	0.759	0.417	3.313	2.136	0.943~4.837	0.069
Working place	0.474	0.185	6.565	1.606	1.118~2.309	0.011
Use of potable water equipment	0.505	0.231	4.779	1.657	1.054~2.606	0.029
Contact history of patients with acute conjunctivitis	0.916	0.352	6.772	2.499	1.254~4.982	0.010
History of chemical substances entering the eyes	0.421	0.264	2.543	1.523	0.908~2.556	0.112
Combined with immune system diseases	0.639	0.388	2.712	1.895	0.886~4.053	0.100
Public toilet utilization rate ≥ 1 times/d	0.642	0.307	4.373	1.900	1.041~3.468	0.037
Washing hand before eating and after toileting	-0.531	0.175	9.207	0.588	0.417~0.829	0.003

Assignment: age (≤40 years old = 1, >40 years old = 0); gender (male = 1, female = 0); working place (outdoor = 1, indoor = 0); use of portable water equipment (yes = 1, no = 0); exposure history of patients with acute conjunctivitis (yes = 1, no = 0); chemical substances into the eye history (yes = 1, no = 0); combined immune system disease (yes = 1, no = 0); public toilet utilization rate ≥ 1 times/d (≥1 times/d = 1, <1 times/d = 0); and washing hands before eating and after toileting (yes = 1, no = 0).

## Data Availability

The labeled dataset used to support the findings of this study is available from the corresponding author upon request.
